The article "lncRNA MRUL Suppressed Non-Small Cell Lung Cancer Cells Proliferation and Invasion by Targeting miR-17-5p/SRSF2 Axis" was retracted in 2024. Reasons: signs of a paper mill; suspected computer-generated content; unreliable results or conclusions; concerns about the data.

# lncRNA MRUL Suppressed Non-Small Cell Lung Cancer Cells Proliferation and Invasion by Targeting miR-17-5p/SRSF2 Axis

**DOI:** 10.1155/2020/9567846

**Published:** 2020-10-07

**Authors:** Ying Chen, Tianle Shen, Xuping Ding, Cui Ma, Lei Cheng, Liming Sheng, Xianghui Du

**Affiliations:** ^1^Department of Radiation Oncology, Zhejiang Key Laboratory of Radiation Oncology, The Cancer Hospital of the University of Chinese Academy of Sciences (Zhejiang Cancer Hospital); Institute of Basic Medicine and Cancer (IBMC), Chinese Academy of Sciences, 1 Banshandong Road, 310022 hangzhou, Zhejiang, China; ^2^Department of Radiation Oncology, Jiaotong University School of Medicine, 197 Ruijin Second Road, 200000 Shanghai, China; ^3^Department of Respiratory Medicine, Affiliated Hangzhou First People's Hospital, Zhejiang University School of Medicine, 310000 Zhejiang, China; ^4^Department of Endocrinology and Metabolism, Zhejiang Greentown Cardiovascular Hospital, 409 Gudun Road, 310000 Zhejiang, China

## Abstract

The two broad histological subtypes of lung cancer are small cell lung cancer (SCLC) and non-small cell lung cancer (NSCLC), which are the leading causes of cancer-related death in the world. Long noncoding RNAs (lncRNAs) have been verified to be critical in the regulation of cancer development. The present study identified and elucidated the regulatory roles of a novel lncRNA MRUL in NSCLC. The results showed that MRUL was overexpressed in NSCLC samples and correlated with the poor prognosis of patients who had NSCLC. Moreover, this research has for the first time demonstrated that MRUL acted as an oncogenetic lncRNA in NSCLC. Knockdown of MRUL considerably repressed NSCLC cell proliferation, invasion, and migration. The bioinformatics analysis showed that MRUL was involved in regulating multiple RNA splicing and proliferation-related biological processes, such as mRNA splicing, RNA splicing, mRNA processing, mRNA 3′-end processing, mRNA splice site selection, and DNA replication. By combining bioinformatics analysis and experimental validation, we found that MRUL regulated NSCLC progression through promoting SRSF2 by sponging miR-17 in NSCLC cells. The discoveries indicated that MRUL could be a therapeutic target and a potential diagnostic for NSCLC.

## 1. Introduction

Lung cancer, which includes small cell lung cancer (SCLC) [1] and non-small cell lung cancer (NSCLC) [2], has been playing the leading part in causing tumor-related death worldwide. NSCLC can then be classified into subcategories of squamous cell carcinoma, adenocarcinoma, and large cell carcinoma [3]. Multiple causes, such as genetic factors, air pollution, and smoking, were regarded to be related to NSCLC progression. However, the mechanisms underlying NSCLC remained to be further investigated.

The article "lncRNA MRUL Suppressed Non-Small Cell Lung Cancer Cells Proliferation and Invasion by Targeting miR-17-5p/SRSF2 Axis" was retracted in 2024. Reasons: signs of a paper mill; suspected computer-generated content; unreliable results or conclusions; concerns about the data.

Long noncoding RNAs (lncRNAs) are a type of ncRNAs which have longer than 200 bps with no or limited protein-coding capacity [4]. Emerging studies demonstrated that lncRNAs participated in regulating cancer tumorigenesis and progression through multiple cancer-related pathways, including Wnt signaling and PI3K signaling. lncRNAs could affect cancer proliferation, differentiation, and metastasis. For example, silencing of PVT1 enhances radiosensitivity in NSCLC by sponging miR-195 [5]. The contribution to NSCLC's progression by lncRNA SNHG1 is made by activating Wnt/*β*-catenin signaling pathway [6] and inhibiting miR-101-3p. And NSCLCAT1 enhanced NSCLC cell migration and invasion via the Hippo signaling pathway through the interaction with CDH1 [7]. Therefore, understanding the roles of lncRNAs in NSCLC is of great significance for exploring the underlying mechanisms of NSCLC progression and discovering new therapeutic strategies for NSCLC.

lncRNA MRUL was a nonprotein coding transcript of DMTF1 [8]. Interestingly, a tumor suppressor as DMTF1 was regarded in human cancers, while MRUL was considered linked with the progression of human cancers. MRUL, for example, in gastric cancer samples, was upregulated, and it was involved in the regulation of multiple drug resistance [9]. Moreover, the functional roles of MRUL in NSCLC remain unknown. This study aimed at figuring out MRUL's expression and role in NSCLC. This study found that in NSCLC tissues, the MRUL expression level was upregulated. Moreover, to explore the potential functions of MRUL in NSCLC, loss-of-function assays were carried out.

## 2. Materials and Methods

### 2.1. The Protein Expression Level of DMTF1 in Lung Cancer Tissues

The Human Protein Atlas (http://www.proteinatlas.org) for the online query was used, DMTF1 was entered in the search field, and the search button was clicked. The option of the lung in the tissue group was selected to evaluate the expression level of DMTF1 protein in lung cancer tissues.

### 2.2. Quantitative Real-Time Polymerase Chain Reaction (qRT-PCR)

TRIzol reagent (Invitrogen, USA) was employed to extract total RNAs from tissues or samples, and the synthesis of cDNA was carried out based on the protocol of the manufacturer. By using SYBR Green qPCR Mixes (Invitrogen, CA) based on the information given by the manufacturer, quantitative real-time PCR (qRT-PCR) was conducted to decide the expression of MRUL and E-cadherin, cyclin D1, N-cadherin, Vimentin, and Snail. Through the use of the IQ5 real-time PCR System machine, qRT-PCR was conducted.

### 2.3. Western Blot Analysis

From cells or tissues, total protein lysates were extracted. By using 10% sodium dodecyl sulfate-polyacrylamide gel electrophoresis (SDS-PAGE), equal quantity of protein was separated, and they were transferred to polyvinylidene difluoride membranes (PVDF, Bio-Rad, Hercules, CA). After blocking with nonfat milk, in the environment of 1 : 3000 dilutions at 4°C overnight, the incubation of membrane with p-AKT and GAPDH antibodies (Bioworld Biotechnology) took place. The incubation of the membrane with secondary antibody (Pierce, IL, USA) was carried out subsequent to its being washed in TBST. The employment of ECL reagents (Pierce, IL, USA) helped to detect the protein band.

The article "lncRNA MRUL Suppressed Non-Small Cell Lung Cancer Cells Proliferation and Invasion by Targeting miR-17-5p/SRSF2 Axis" was retracted in 2024. Reasons: signs of a paper mill; suspected computer-generated content; unreliable results or conclusions; concerns about the data.

### 2.4. Cell Lines, Cell Cultures, and Transfections

The Academy of Military Medical Sciences (Beijing, China) provided the human NSCLC cell line A549 and H1299. In a 5% CO_2_ humidified incubator at 37°C and RPMI 1640 medium (Thermo Scientific, USA) supplemented with 10% fetal calf serum (FCS) (Thermo Scientific), these cells were cultured. For transfections, pcDNA3.1(+)-MRUL and pcDNA3.1(+) vector (DingGuoChangSheng Biotechnology Co. Ltd., Beijing, China), 50 to 100 nM small interfering RNA (siRNA) (Gene Pharma Co., Shanghai, China), Lipofectamine 2000 (Invitrogen Int., USA), and lentivirus vector-MRUL(−) (RiboBio Co., Guangzhou, China) were employed following the manufacturer's recommendations as portrayed earlier (19). siRNA sequences are presented here: siRNA targeting NR_024549 (MRUL), siMRUL-1, GGCCUUUGUUUGCAGUUUATT; siMRUL-2, AACACUUUCCUGUUUUGGGUC; siMRUL-3, AGUUUCUACUGUUACUGUGUC; siP-gp (targeting P-gp), GGGACAGGAAUAAUUAUAUTT; and siNC (negative control), UUCUCCGAACGUGUCACGUTT.

### 2.5. Cell Growth and Invasion

To assay cell growth, the incubation of the cells happened in the 96-well plate, and they were stained with CCK-8 (Dojindo Chemical Laboratory, Kumamoto, Japan) at different moments. The multilabel plate reader (PerkinElmer, MA) was employed to decide the absorbance at 450 nm. Matrigel-coated Transwell chambers (Millipore, MA, USA) helped to measure cell invasion. On the upper chamber where no serum existed, those cells were cultured. In the bottom well, the medium with 10% FBS was added to make it the chemoattractant. One percent crystal violet was used to fix the invasive cells, and then, they were counted.

### 2.6. Statistical Analysis

All of the results were presented as mean ± standard deviation (SD). All experiments were repeated at least 3 times, and representative experiments were shown. SPSS [10] statistical (SPSS, Chicago, USA) was employed to conduct statistical analysis. Student's *t*-test analysis of variance was employed to measure the statistical difference. If *p* is below 0.05, then the difference was considered statistically significant.

The article "lncRNA MRUL Suppressed Non-Small Cell Lung Cancer Cells Proliferation and Invasion by Targeting miR-17-5p/SRSF2 Axis" was retracted in 2024. Reasons: signs of a paper mill; suspected computer-generated content; unreliable results or conclusions; concerns about the data.

## 3. Result

### 3.1. The RNA Levels, Not Protein Levels of DMTF1 Expression, Were Increased in NSCLC Samples

lncRNA MRUL was a nonprotein coding transcript of DMTF1. DMTF1 was reported to be a tumor suppressor. Very interestingly, we found that DMTF1 RNA levels were significantly upregulated in both types of NSCLC samples, including LUAD and LUSC tissues by analyzing the TIMER database (Figure 1(a)), suggesting that DMTF1 might serve as an oncogene in NSCLC, and this did not go along with past studies.

Furthermore, we analyzed the protein levels of DMTF1 in NSCLC using The Human Protein Atlas. The results showed that DMTF1 protein levels were not significantly dysregulated in lung cancer samples compared to normal tissues. Thus, we hypothesized that DMTF1 played its roles in NSCLC probably via its nonprotein coding transcripts. What is more, the association between lower expression levels of lncRNA MRUL and advanced stage in patients who had NSCLC had been discovered (Figure 1(b)).

### 3.2. High lncRNA MRUL Expression Correlates with Poor Survival of LUAD but Not LUSC

To explore whether the relation between lncRNA MRUL and the survival of patients who had lung cancer existed, we performed the Kaplan-Meier curve analysis by using the TCGA database. As presented in Figure 2, it was found the positive correlation existed between higher lncRNA MRUL expression and shorter disease-free survival time in patients who had LUAD (Figure 2(a)), but not LUSC (Figure 2(b)), indicating that lncRNA MRUL might be a biomarker of poor survival. Furthermore, the Kaplan-Meier plotter database was employed to analyze the association between lncRNA MRUL expression and the prognosis. An amount of 1926 cases of NSCLC together with available data for lncRNA MRUL expression and the general rate of survival were included in the database.

This study showed that higher lncRNA MRUL expression was associated with shorter first progression survival time and overall survival time in LUAD, but not with LUSC (Figures 2(c)–2(e)). Similar results were also observed by analyzing an independent GEO dataset, GSE50081 (Figures 2(f)–2(h)).

### 3.3. Knockdown of lncRNA MRUL Suppressed NSCLC Cell Proliferation and Cell Cycle

This study further teased out the subcellular localization of MRUL in NSCLC cells, including A549 and H1299 cells. The RT-PCR assay results made it clear that compared with the MRUL level in nuclear in both H1299 and A549 cell lines, it was higher in the cytoplasm (Figures 3(a) and 3(b)), suggesting that MRUL was a cytoplasm located in lncRNA. In order to work out MRUL's functional effect on NSCLC cell, 2 siRNAs reported by previous studies were used to knockdown the expression levels of MRUL in H1299 and A549 cells. The knockdown efficiency was presented in (Figures 3(c) and 3(d)).

The article "lncRNA MRUL Suppressed Non-Small Cell Lung Cancer Cells Proliferation and Invasion by Targeting miR-17-5p/SRSF2 Axis" was retracted in 2024. Reasons: signs of a paper mill; suspected computer-generated content; unreliable results or conclusions; concerns about the data.

In an effort to detect MRUL's effect on cell proliferation, the CCK-8 assays were applied (Figures 3(e)–3(h)). We noticed that compared with siNC transfected cells, the cell viability decreased considerably in siMRUL-1- and siMRUL-2-transfected cells. The flow cytometric analysis made it clear that the knockdown of MRUL significantly increased the proportion of G1 phase cells by 30% and reduced the proportion of S phase cells by 30%. These results suggested MRUL played as an oncogene in NSCLC.

### 3.4. Knockdown of lncRNA MRUL Suppressed NSCLC Cell Migration and Invasion

This study then looked at whether NSCLC cell invasion and migration abilities were affected by MRUL. Through the performance of Transwell assay, we found the migrating cells in siMRUL-1- and siMRUL-2-transfected A549 cells decreased by about 62 and 56 percentage compared to control groups (Figures 4(a) and 4(b)). By adding Matrigel in a Transwell chamber, this study further detected the influence on the invasive ability of NSCLC produced by MRUL knockdown. The results suggested that MRUL knockdown significantly inhibited A549 cell invasion. The numbers of invading cells decreased by 36 and 41.3 percentage in siMRUL-1- and siMRUL-2-transfected A549 cells, compared with control groups (Figures 5(a) and 5(b)). The results obtained by using H1299 cells were also similar (Figures 4(c), 4(d), 5(c), and 5(d)).

### 3.5. Functional Analysis of lncRNA MRUL in NSCLC

The detailed mechanisms of MRUL regulating NSCLC progression remained largely unclear. Here, we conducted a coexpression analysis of MRUL in NSCLC using the cBioPortal database [11] (https://www.cbioportal.org/). After selection, the potential targets of MRUL in NSCLC were the top 1000 coexpressing genes. GO analysis of the 1000 target genes revealed that some of the biological processes were involved, such as transcription, mRNA splicing, RNA splicing, mRNA processing, mRNA 3′-end processing, RNA processing, regulation of protein kinase activity, cilium morphogenesis, mRNA splice site selection, regulation of RNA splicing, DNA replication, cilium-dependent cell motility, cilium assembly, RNA export from the nucleus, and mismatch repair (Figure 6(a)).

Furthermore, the PPI [12] network revealed interactions between target genes (Figure 7(a)). The use of the MCODE plugin (the nodes with edges ≥ 2 − core and degree cut − off ≥ 2) helped perform module analysis, and we identified four hub networks regulated by MRUL in NSCLC. Figures 6(b)–6(e) show that there are 68 edges and 19 nodes in hub network 1, 37 edges and 13 nodes in hub network 2, 16 edges and 10 nodes in hub network 3, and 13 edges and 9 nodes in hub network 4.

The article "lncRNA MRUL Suppressed Non-Small Cell Lung Cancer Cells Proliferation and Invasion by Targeting miR-17-5p/SRSF2 Axis" was retracted in 2024. Reasons: signs of a paper mill; suspected computer-generated content; unreliable results or conclusions; concerns about the data.

Next, the potential functions of these hub networks in NSCLC were disclosed through the application of the ClueGO [13] analysis. These results showed the involvement of hub network 1 in regulating the termination of RNA polymerase II transcription, spliceosome, and mRNA splicing. Hub network 2 was involved in regulating centriole. These results were consistent with the above analysis that lncRNA MRUL was associated with the regulation of RNA splicing Figures 7(a) and 7(b).

### 3.6. MRUL Regulated SRSF2 Expression

The bioinformatics analysis showed the involvement of MRUL in regulating RNA splicing and cell cycle. In order to validate these findings, we knocked down lncRNA MRUL expression and detected RNA splicing regulators expression in NSCLC cell, including RBM25, RBM39, RBM5, RNPC3, SUGP2, THOC1, ACIN1, PRPF3, PRPF38B, PRPF4B, SRSF11, and SRSF2 **(**Figure 8(a)). The results showed that knockdown of MRUL significantly suppressed SRSF11, SRSF2, RBM25, RBM39, and RBM5 expression in A549 and H1299 cells. Among these regulators, the inhibition of SRSF2 expression was the most significant; we focused on SRSF2, which was taken as an oncogene in human cancers and involved in regulating cell cycle and metastasis. By detecting the protein levels of SRSF2 after silencing of MRUL, the results showed knockdown of MRUL inhibited SRSF2 protein levels **(**Figures 8(b) and 8(c)).

### 3.7. MRUL Regulated SRSF2 Expression via Physically Binding to miR-17-5p

Next, we predicted the miRNAs targeting MRUL regulated SRSF2 using the miRDB database (http://mirdb.org/). A total of 20 candidate miRNAs were identified to target both MRUL and SRSF2 (Figure 9(a)). Then, we compared them based on their predicted scores and free energy. These miRNAs were prioritized, and miR-17-5p was selected for subsequent analysis. This study was centered on miR-17-5p, which was reported as a tumor suppressor. The correlation analysis showed the expression levels were negatively correlated to the expression levels of MRUL (Figures 9(g) and 9(h)) and SRSF2 (Figures 9(b) and 9(c)). Enhanced expression of miR-17-5p considerably suppressed the luciferase activity of constructed reporter containing MRUL and SRSF2, but not the empty reporter, which has been displayed by the dual-luciferase reporter assays. RT-PCR assays showed that SRSF2 and MRUL levels in both A549 and H1299 cells were suppressed by overexpression of miR-17-5p (Figures 9(f) and 9(i)). Enhanced expression of miR-17-5p suppressed SRSF2 protein levels in both A549 and H1299 cells, which was displayed by Western blot assays (Figures 9(d) and 9(e)).

The article "lncRNA MRUL Suppressed Non-Small Cell Lung Cancer Cells Proliferation and Invasion by Targeting miR-17-5p/SRSF2 Axis" was retracted in 2024. Reasons: signs of a paper mill; suspected computer-generated content; unreliable results or conclusions; concerns about the data.

## 4. Discussion

Recently, emerging evidences demonstrated that lncRNAs were deregulated and played crucial roles in tumor tumorigenesis and pathogenesis. In NSCLC, a series of lncRNAs were reported to be related to cancer progression. For example, via suppressing autophagy, the chemosensitivity of NSCLC cells is enhanced by silencing lncRNA-XIST, and through regulating the WNT pathway in NSCLC and repressing E-cadherin, epithelial-mesenchymal transition (EMT) is enhanced by the overexpression of FEZF1-AS1 [14]. The present study identified and elucidated the regulatory roles of a novel lncRNA MRUL in NSCLC. The results showed that MRUL was overexpressed in NSCLC samples and correlated with the poor prognosis of NSCLC patients. Moreover, this research for the first time demonstrated MRUL played as an oncogenetic lncRNA in NSCLC. NSCLC cell proliferation, invasion, and migration were considerably suppressed by the knockdown of MRUL. By combining bioinformatics analysis and experimental validation, we found that MRUL regulated NSCLC progression through promoting SRSF2 by sponging miR-17 in NSCLC cells. These results suggested the potential of MRUL to be a diagnostic and therapeutic target of NSCLC.

DMTF1 was regarded as a tumor suppressor in human cancers [15]. DMTF1 was regulated by Ras-Raf signaling and involved in activating the Arf-p53 pathway [16]. Previous studies reported that in roughly 40% of human NSCLC samples, the DMTF1 gene was deleted [17]. However, for tumor suppression in Kras-mediated lung carcinogenesis mouse models, DMTF1 is haplo-insufficient [18]. Very interestingly, through the analysis of public datasets, which include the LUAD, TCGA [19], and LUSC databases, this study found that compared with normal tissues, DMTF1 RNA levels were significantly overexpressed in NSCLC samples. Importantly, protein levels of DMTF1 in NSCLC were not remarkably dysregulated. These results suggested DMTF1 might play its roles in NSCLC via its nonprotein coding transcripts. lncRNA MRUL was a nonprotein coding transcript of DMTF1. A previous study revealed that MRUL was involved in regulating multidrug-resistance in gastric cancer (GC) cell via ABCB1 [20]. Compared with normal tissues, MRUL was considerably overexpressed in GC. MRUL knockdown in GC cells promoted cell apoptosis [21]. Nevertheless, MRUL's roles in NSCLC remain to be classified. This study made it clear that compared with early-stage NSCLC samples, lncRNA MRUL was overexpressed in advanced stage NSCLC samples. Higher expression levels of MRUL were significantly correlated with shorter disease-free survival time in patients with LUAD, but not LUSC, which has been shown in the Kaplan-Meier curve analysis. Moreover, knockdown of lncRNA MRUL decreased NSCLC cell cycle, cell growth, invasion, and migration. In sum, the data indicated that lncRNA MRUL was probably an oncogene in NSCLC.

The article "lncRNA MRUL Suppressed Non-Small Cell Lung Cancer Cells Proliferation and Invasion by Targeting miR-17-5p/SRSF2 Axis" was retracted in 2024. Reasons: signs of a paper mill; suspected computer-generated content; unreliable results or conclusions; concerns about the data.

Aiming to investigate the detailed mechanisms of MRUL in NSCLC, we applied the GO and KEGG pathway analysis and coexpression analysis for MRUL. The bioinformatics analysis showed that MRUL was involved in regulating multiple RNA splicing and proliferation-related biological processes, such as mRNA splicing, RNA splicing, mRNA processing, mRNA 3′-end processing, mRNA splice site selection, and DNA replication. By constructing PPI networks, we identified the critical role of SRSF2 in MRUL regulating networks and its involvement in regulating RNA splicing in cancer progression. Furthermore, we found that knockdown of MRUL significantly suppressed SRSF2 expression in NSCLC cells. SRSF2 is a gene encoding a key spliceosome protein and a key regulator of RNA splicing disorders in cancer. Related reports have shown that SRSF2 is essential for the pathogenesis and progression of liver cancer cells and can be used as a prognostic factor for HCC patients. In clear cell renal cell carcinoma, decreased expression of SRSF2 contributes to the protection of cancer cell viability. By using bioinformatics analysis, we predicted that lncRNA's effect upon MRUL expression was mediated by miR-17-5p. Further validation showed that MRUL and SRSF2 were miR-17-5p's direct targets. Being a member of miR-17-92 cluster, miR-17-5p played as a key regulator of cancer proliferation, cell cycle, apoptosis, and autophagy. The expression of miR-17-5p is upregulated in pancreatic adenocarcinoma, and high levels of miR-17-5p are associated with poor prognosis. It was found in colon cancer that miR-17-5p reduced the expression of tumor suppressor B cell junction (BLNK), leading to increased migration and invasion of cancer cells. In NSCLC, emerging evidences demonstrated miR-17-5p functioned as a potential biomarker for cancer prognosis and a tumor suppressor. It was found that miR-17-5p was downregulated in NSCLC, and the negative relation between serum miR-17-5p levels and the survival of NSCLC patients was also discovered. Mechanically, miR-17-5p suppressed multiple targets in NSCLC, including BECN1, RAD21, STAT3, and lncRNA H19. SRSF2 was reported to regulate gene splicing and alternative splicing [22]. SRSF2 acted as an oncogene and regulated transcriptional extension and activation, and by interacting with E2F1 [23], it stimulated gene-regulated cell cycle activity. In NSCLC, SRSF2 could enhance cancer proliferation by regulating VEGFR1 pre-mRNA alternative splicing [24].

The article "lncRNA MRUL Suppressed Non-Small Cell Lung Cancer Cells Proliferation and Invasion by Targeting miR-17-5p/SRSF2 Axis" was retracted in 2024. Reasons: signs of a paper mill; suspected computer-generated content; unreliable results or conclusions; concerns about the data.

More and more evidence show that lncRNAs can be used as ceRNAs and can regulate the expression of mRNAs by binding to miRNAs. The function of lncRNA is closely related to its subcellular location. In this study, we determined that MRUL is mainly located in the cytoplasm of lung cancer cells, suggesting that MRUL may be an endogenous miRNA sponge. Bioinformatics analysis and luciferase report analysis indicate that MRUL and SRSF2 are direct targets of miR-17-5p. In addition, overexpression of miR-17-5p inhibits the expression levels of SRSF2 and MRUL, and enhanced expression of miR-17-5p inhibits the level of SRSF2 protein in cells. These data indicate that there may be a regulatory mechanism in lung cancer tissues. MRUL competitively sponges miR-17-5p to regulate the expression of SRSF2 mRNA, and miR-17-5p mediates between MRUL and SRSF2. Overexpression of MRUL in lung tumors can absorb more miR-17-5p, which leads to miR17-5p reducing miRNA-mediated SRSF2 mRNA attenuation, thereby promoting the aggressive growth of tumors and ultimately affecting patient survival.

In conclusion, lncRNA MRUL expression was upregulated in NSCLC tissues. We have demonstrated for the first time that MRUL acts as an oncogenic regulator in NSCLC and promotes cell proliferation and metastasis. Partly through regulating the miR-17-5p/SRSF2 pathway in NSCLC, lncRNA MRUL knockdown suppressed cell growth, migration, and cell invasion. The outcome produced by this study indicated the potential of lncRNA MRUL to be a biomarker and a valuable target for therapies in NSCLC.

## Figures and Tables

**Figure 1:** Long noncoding RNA MRUL was upregulated in NSCLC. (a) MRUL expression levels were downregulated in LUAD and LUSC samples compared with normal tissues. (b) The protein levels of DMTF1 were not significantly dysregulated in NSCLC samples compared to normal lung tissues. Significance was defined as *p* < 0.05 (∗*p* < 0.05; ∗∗*p* < 0.01; ∗∗∗*p* < 0.001).

**Figure 2:** High lncRNA MRUL expression correlates with poor survival of LUAD, but not LUSC. (a, b) TCGA dataset analysis revealed that high lncRNA MRUL expression correlates with poor survival of LUAD, but not LUSC. (c–e) The Kaplan-Meier plotter database analysis revealed high lncRNA MRUL expression correlated with poor survival of NSCLC and LUAD, but not LUSC. (f–g) GSE50081 dataset analysis revealed that high lncRNA MRUL expression correlated with poor survival of NSCLC and LUAD, but not LUSC. Significance was defined as *p* < 0.05 (∗*p* < 0.05; ∗∗*p* < 0.01; ∗∗∗*p* < 0.001).

**Figure 3:** Knockdown of lncRNA MRUL suppressed NSCLC proliferation. (a, b) RT-PCR assay showed MRUL was located in the cytoplasm in both A549 and H1299 cells. (c, d) RT-PCR assay showed MRUL expression levels in A549 and H1299 cells after transfecting with siRNA-1 and siRNA-2. (e, f) Knockdown of MRUL induced cell proliferation in A549 and H1299. Significance was defined as *p* < 0.05 (∗*p* < 0.05; ∗∗*p* < 0.01; ∗∗∗*p* < 0.001).

The article "lncRNA MRUL Suppressed Non-Small Cell Lung Cancer Cells Proliferation and Invasion by Targeting miR-17-5p/SRSF2 Axis" was retracted in 2024. Reasons: signs of a paper mill; suspected computer-generated content; unreliable results or conclusions; concerns about the data.

**Figure 4:** Knockdown of MRUL induced cell migration in NSCLC. (a, b) Knockdown of MRUL suppressed cell migration ability in A549 cells. (c, d) Knockdown of MRUL suppressed cell migration ability in H1299 cells. Significance was defined as *p* < 0.05 (∗*p* < 0.05; ∗∗*p* < 0.01; ∗∗∗*p* < 0.001).

**Figure 5:** Knockdown of MRUL induced cell invasion in NSCLC. (a, b) Knockdown of MRUL suppressed cell invasion ability in A549 cells. (c, d) Knockdown of MRUL suppressed cell invasion ability in H1299 cells. Significance was defined as *p* < 0.05 (∗*p* < 0.05; ∗∗*p* < 0.01; ∗∗∗*p* < 0.001).

**Figure 6:** Bioinformatics analysis of MRUL in NSCLC. (a) Bioinformatics analysis of MRUL in NSCLC. (b–e) Construction of hub networks regulated by MRUL in NSCLC, including hub network 1 (b), hub network 2 (c), hub network 3 (d), and hub network 4 (e).

**Figure 7:** Bioinformatics analysis of MRUL regulated hub networks 1 and 2 in NSCLC. (a, b) Bioinformatics analysis of MRUL regulated hub networks 1 (a) and 2 (b) in NSCLC.

**Figure 8:** Validation of downstream targets of MRUL. (a) RT-PCR assay showed the expression levels of downstream targets after transfecting with siMRULs. (b, c) Western blot assay revealed the protein levels of SRSF2 after transfecting with siMRULs in A549 (b) and H1299 (c).

**Figure 9:** MRUL regulated SRSF2 expression via physically binding to miR-17-5p. (a) Venn diagrams for SRSF2-binding miRNAs and MRUL-binding miRNAs. (b, c) RT-PCR analysis of SRSF2 expression levels in A549 and H1299 after transfecting with miR-17-5p mimics. (d, e) Western blot analysis of SRSF2 protein levels in A549 and H1299 after transfecting with miR-17-5p mimics. (f) Luciferase assay detects the direct binding of miR-17-5p on the 3-UTR of SRSF2. (g, h) RT-PCR analysis of MRUL expression levels in A549 and H1299 after transfecting with miR-17-5p mimics. (i) Luciferase assay detects the direct binding of miR-17-5p on the MRUL.

## Data Availability

The datasets used and/or analyzed during the current study are available from the corresponding author on reasonable request.
